The article "Effect of Loratadine Tablets in Combination with Other Drugs on Nasal Physiological Function and T Lymphocyte Subsets in Patients with Allergic Rhinitis" was published in 2022. Journal: Comput Intell Neurosci.

# Effect of Loratadine Tablets in Combination with Other Drugs on Nasal Physiological Function and T Lymphocyte Subsets in Patients with Allergic Rhinitis

**DOI:** 10.1155/2022/3990427

**Published:** 2022-08-21

**Authors:** Jie Zhang, Hongzheng Cheng, Yi Luo, Dan Kan, Yinghuai Wang

**Affiliations:** PuRen Hospital Affiliated to Wuhan University of Science and Technolog/Otorhinolaryngology, No. 1 Benxi Street, Qingshan District, Wuhan City 430081, Hubei Province, China

## Abstract

**Objective:**

To investigate the effects of loratadine tablets in combination with other drugs on nasal physiological function and T lymphocyte subsets in patients with allergic rhinitis (AR).

**Methods:**

A total of 120 AR patients treated in our hospital from February 2018 to February 2021 were randomly divided into control group and research group. The control group was given mometasone furoate nasal spray combined with loratadine tablets, while the research group was given budesonide combined with loratadine. The efficacy, duration of clinical symptom remission, immune function indicators, T lymphocyte subset, nasal physiological function, and incidence of adverse reactions were compared between the two groups.

**Results:**

The efficacy results of the two groups showed that the effective rate of the research group was 96.67%, while the effective rate of the control group was 83.33%. The effective rate in the research group was higher compared to the control group (*χ*^2^: 5.925 *P* < 0.05). The results of clinical symptom relief time showed that the clinical symptom relief time of nasal congestion, itching, runny nose, and sneezing in the research group was lower than that in the control group, and the difference was statistically significant (*P* < 0.05). The results of the comparison of immune function indicators showed that the IL-6, IL-8, and IgE of the research group were lower than those of the control group, while the Th1/Th2 of the research group were higher than those of the control group. There were no statistically significant differences in T lymphocyte subsets before nursing, but after treatment, the T lymphocyte subsets of the two groups decreased, and the level of CD3+, CD4+, CD8+, CD4+, and CD4+/CD8+ lymphocytes in the research group was lower than that of the control group, and the difference was statistically significant (*P* < 0.05). Before treatment, there exhibited no significant difference in nasal physiological function, but after treatment, the nasal physiological function of the two groups was enhanced, and the MTT, NR, and MCR of the research group were lower than those of the control group, and the difference was statistically significant (*P* < 0.05). Finally, the incidence of adverse reactions in the research group was lower compared to the control group, and the difference was statistically significant (*P* < 0.05).

The article "Effect of Loratadine Tablets in Combination with Other Drugs on Nasal Physiological Function and T Lymphocyte Subsets in Patients with Allergic Rhinitis" was published in 2022. Journal: Comput Intell Neurosci.

**Conclusion:**

Budesonide and loratadine are effective in improving patient efficacy, T lymphocyte subsets, and nasal physiological function, and are safer.

## 1. Introduction

Allergic rhinitis (AR) is an IgE-mediated noninfectious disease of nasal mucosa characterized by the activation and infiltration of inflammatory cells [1]. The main inflammatory cells involved are mast cells and eosinophils. The main clinical symptoms of AR are nasal blockage, runny nose, nasal itching, and sneezing. Some patients are also accompanied by itching and tears, which are mainly seen in patients with AR caused by pollen [2]. The main clinical symptoms are runny nose, nasal congestion, paroxysmal sneezing, nasal itching, sleep and breathing disorders, otitis media, sinusitis, and other complications [3]. When patients with AR are exposed to allergens such as dust mites, the immune response starts, and the immune response tends to develop in the direction of Th2 type immune response, which promotes Th2 cells to secrete allergy-related cytokines. These inflammatory factors further promote B cells to secrete antigen-specific IgE (sIgE). When the allergen restimulates the immune process of the body, sIgE binds quickly to the allergen epitope and crosslink occurs, which makes mast cells degranulate and release allergic and inflammatory mediators, damage nasal mucosa and lead to AR [4].

Oxidative stress injury also plays an important role in the pathogenesis of AR [5]. Oxidative stress and related inflammatory pathways are mainly regulated by nuclear factor E2-related factor 2 (Nrf2)/heme oxygenase-1 (HO-1) pathway and NF-*κ*B signal pathway [6]. When Nrf2 binds to its corresponding inhibitory protein, ubiquitin degradation leads to a decrease in its activity. When the body is subjected to stress, reactive oxygen species can make nuclear factor E2-related factor 2 enter the nucleus, initiate HO-1 transcription and expression, inhibit NF- *κ* B signal pathway, and play an antioxidant role [7]. Regulatory T cells (Treg) are a class of T cells that express CD4, CD25, and transcription factor Foxp3. They dynamically regulate immune homeostasis by regulating Th1/Th2 balance. Some studies have indicated that the levels of IL-4 and effector T cells in patients with allergic diseases are significantly higher compared to patients without allergic diseases, while the levels of IL-10 and Treg are decreased [8]. Adoptive transfer of Treg cells can prevent or alleviate autoimmune diseases, resulting in immune tolerance to allergens [9]. Therefore, strengthening the level of Treg is an important strategy in the treatment of AR. Avoiding contact with allergens is still the main means of prevention and treatment of AR.

The article "Effect of Loratadine Tablets in Combination with Other Drugs on Nasal Physiological Function and T Lymphocyte Subsets in Patients with Allergic Rhinitis" was published in 2022. Journal: Comput Intell Neurosci.

Loratadine tablets were often employed to treat children in the past [9]. Loratadine belongs to the second generation of antihistamine drugs, which play a good antiallergic effect mainly by inhibiting the binding of histamine to H1 receptor [10]. However, some studies have proved that the effect of loratadine alone in the treatment of AR has some limitations, and it is easy to relapse after drug withdrawal [11]. Based on this, it is necessary to explore other adjuvant treatments. A large number of studies have demonstrated that glucocorticoid has good anti-inflammatory and antiallergic effects, can significantly reduce a variety of inflammatory reactions, and alleviate nasal allergy [12]. Existing treatments or drugs can only relieve the symptoms of AR and need long-term medication, and adverse reactions caused by existing therapeutic drugs are constantly reported, such as liver and gastrointestinal diseases, lethargy, jaundice, nasal irritation, rashes, diarrhea, and so on. Meanwhile, the period of immunotherapy is long, the compliance of patients is poor, the treatment results vary greatly, and the treatment effect is not ideal. Therefore, it is necessary to actively explore an effective scheme for the treatment of patients. In the past, loratadine was often employed to treat children, although it has a certain effect but the overall effect needs to be enhanced [12]. Mometasone furoate nasal spray combined with loratadine, budesonide and loratadine can achieve good results in the treatment of AR, but there are few reports on the clinical efficacy of the two regimens in the treatment of AR. Therefore, in this study, the aim is to explore the efficacy of different drugs combined with loratadine tablets in the treatment of AR and the effects of T lymphocyte subsets and nasal physiological function.

## 2. Patients and Methods

### 2.1. General Information

One hundred and twenty patients with AR treated in our hospital from February 2018 to February 2021 were enrolled. The patients were randomly assigned into a control group and a research group. The control group was treated with mometasone furoate nasal spray combined with loratadine tablets, and the research group was treated with budesonide and loratadine. In the control group, the age was 18–74 years old, with an average of (45.66 ± 3.31) years, including 32 males and 28 females, while in the research group, the age was 18–76 years old, with an average of (45.33 ± 3.44) years, including 36 males and 24 females. There exhibited no statistical significance in the general data of the two groups. This study was permitted by the Medical Ethics Association of our hospital, and all patients signed informed consent.

The article "Effect of Loratadine Tablets in Combination with Other Drugs on Nasal Physiological Function and T Lymphocyte Subsets in Patients with Allergic Rhinitis" was published in 2022. Journal: Comput Intell Neurosci.

Diagnostic criteria: according to the relevant diagnostic criteria mentioned in the clinical guidelines for allergic rhinitis issued by the American Society of Otorhinolaryngology and head and neck surgery in 2014 [13]: (1) there are two or more main symptoms such as nasal congestion, nasal itching, sneezing, and runny nose in clinic. The cumulative time of the symptoms may be more than 1 hour, and there can be both eye symptoms such as itching, conjunctival congestion, tears, and so on; (2) there are common watery secretions in the nasal cavity with edema and pallor of the nasal mucosa; and (3) the clinical manifestation of allergic rhinitis should be consistent with the results of skin prick test or serum specific IgE test.

Inclusion criteria: those who meet all of the following items can be included. (1) Patients, who meet the above diagnostic criteria; (2) 18 years old ≤ age ≤80 years old; (3) the total score of nasal symptoms (TNSS) ≥4; and (4) voluntarily participate in this study and sign the informed consent form for treatment.

Exclusion criteria: those, who meet any of the following items cannot be included. (1) Those who have taken H1-antihistamines, steroids, AH, decongestants directly acting on the eyes, nose and mouth, corticosteroids, antibiotics, and other drugs within 14 days before treatment; those who have received SLIT, SCIT immunotherapy, or hormone system therapy in the last year. Those, who received physiotherapy in traditional Chinese medicine and other traditional Chinese medicine fields such as acupuncture, moxibustion, cupping, inhalation of traditional Chinese medicine and other traditional Chinese medicine within 14 days before treatment; those who had taken proprietary medicine or decoction that had a significant effect on AR within 14 days before treatment, or those who could not be treated with acupuncture; (2) other types of rhinitis not caused by AR, such as runny nose, stuffy nose, sneezing, itching and ant sensation; (3) patients with respiratory infection within 14 days before enrollment, chronic paranasal sinusitis in previous history or chronic paranasal sinusitis demonstrated by X-ray examination of paranasal sinuses, nasal polyps, severe deviation of nasal septum, severe organic lesions in nasal cavity or undergoing surgery, patients with a history of respiratory diseases; (4) Asthma or vasomotor rhinitis; (5) Serum aspartate aminotransferase (AST), alanine aminotransferase (ALT), creatinine and cystatin C (CysC) >1.5 times the upper limit of normal value; (6) there are serious primary diseases such as cardiovascular, liver, kidney, lung and blood, or serious diseases such as tumor and AIDS; (7) pregnant, lactating women, or persons with physical and mental disabilities; (8) by asking patients to identify those, who have used alcohol, hormone drugs and other medical history, or through the analysis of researchers, the probability of joining the group is low and the situation of joining the group is complicated; (9) patients, who have recently participated in other clinical drug studies; (10) there are people, who are allergic to the ingredients used in this study; and (11) those, who have joined the clinical trials of drugs in the past three months.

The article "Effect of Loratadine Tablets in Combination with Other Drugs on Nasal Physiological Function and T Lymphocyte Subsets in Patients with Allergic Rhinitis" was published in 2022. Journal: Comput Intell Neurosci.

### 2.2. Treatment Methods

The control group was treated with loratadine (trade name: Kai Ruitan, Bayer Pharmaceutical Co., Ltd. (Shanghai), Chinese medicine: H10970410 10 mg/tablet, 6 tablets/box), one tablet at a time, once a day. Budesonide nasal spray (specification: 64 ug^∗^120 sprays; nasal preparation; approval number: national drug standard J20180023; manufacturer: Sweden AstraZenecaAB) was treated twice a day at a dose of 64 ug.

The research group was treated with mometasone furoate nasal spray combined with loratadine tablets, and the treatment method of loratadine tablets was the same as that of the control group. In addition, patients were sprayed with mometasone furoate nasal spray per nostril (manufacturer: Schering-PloughLaboN.V. (Belgium), approval number: H20140100), once a day. Patients in both groups were treated continuously for 1 month.

### 2.3. Observation Index

#### 2.3.1. Curative Effect Evaluation

The criteria for evaluating the curative effect are as follows: effective: after treatment, the symptoms such as sneezing, nasal itching, and runny nose disappeared, and the nasal secretion specific IgE test was negative; effective: after treatment, the symptoms such as sneezing, nasal itching, and runny nose were significantly relieved, and the nasal secretion specific IgE test was negative. Ineffective: after treatment, the symptoms such as sneezing, nasal itching, and runny nose were not significantly enhanced, and the specific IgE test of nasal secretions was negative and positive. Total effective rate = (number of effective cases + number of effective cases)/total number of cases × 100%.

#### 2.3.2. Clinical Symptom Relief Time

Statistics of the two groups of patients with a stuffy nose, nasal itching, runny nose, and sneeze clinical symptoms relief time.

#### 2.3.3. Detection of Immune Function Index

In the early morning fasting state, after EDTA anticoagulation treatment, 3000 rpm, centrifugation 10 min, the upper serum was frozen at −80°C to be tested. The levels of IL-6, IL-8, IgE, and Th1/Th2 in serum were examined by enzyme-linked immunosorbent assay (ELisa). All the kits are obtained from Redd Company of the United States and operate strictly in accordance with the standards of the instructions. The intrabatch differences are less than 10% and the interbatch differences are less than 15%.

The article "Effect of Loratadine Tablets in Combination with Other Drugs on Nasal Physiological Function and T Lymphocyte Subsets in Patients with Allergic Rhinitis" was published in 2022. Journal: Comput Intell Neurosci.

#### 2.3.4. T Lymphocyte Subsets Level

T lymphocyte subsets level: all patients employed EDTA-K2 anticoagulant tube to collect peripheral venous blood 2 mL under the condition of fasting in the morning, then stained with corresponding fluorescence-labeled monoclonal antibody, incubated 30 min at room temperature without light, employed FACSLysingsolusion for hemolysis, and examined the levels of CD3+, CD4+, CD8+, and CD4+/CD8+ lymphocytes by flow cytometry.

#### 2.3.5. Physiological Function of Nasal Cavity

Nasal physiological functions include nasal resistance (NR), nasal mucosal ciliary transit time (MTT), and nasal mucosal ciliary clearance rate (MCR). NR was examined by nasal resistance meter (manufacturer: GM, UK, model: NR6). The detection methods of MTT and MCR were saccharin clearance tests.

#### 2.3.6. Incidence of Adverse Reactions

The incidence of adverse reactions in the two groups was calculated.

### 2.4. Statistical Analysis

SPSS23.0 statistical software was adopted to process the data. The measurement data were presented as ($\bar{x}\pm s$). The group design *t*-test was adopted for the comparison and the analysis of variance was adopted for the comparison between multiple groups. Dun-net-t test was adopted for comparison with the control group. The counting data were presented in the number of cases and the percentage, *χ*^2^ test was adopted for comparison between groups, and a bilateral test was employed for all statistical tests.

## 3. Results

### 3.1. Comparison of Curative Effect

First of all, we compared the curative effects of the two groups: the research group was significantly effective in 36 cases, effective in 22 cases, ineffective in 2 cases, the effective rate was 96.67%; in the control group, 23 cases were significantly effective, 27 cases were effective, 10 cases were ineffective, and the effective rate was 83.33%. The effective rate in the research group was higher compared to the control group (*χ*^2^: 5.925 *P* < 0.05). All the data results are indicated in Figure 1.

### 3.2. Comparison of Clinical Symptom Relief Time

Secondly, we compared the clinical symptom relief time. The clinical symptom relief time of stuffy nose, itching, runny nose, and sneezing in the research group were lower compared to the control group, and the difference was statistically significant (*P* < 0.05). All the data results are indicated in Table 1.

The article "Effect of Loratadine Tablets in Combination with Other Drugs on Nasal Physiological Function and T Lymphocyte Subsets in Patients with Allergic Rhinitis" was published in 2022. Journal: Comput Intell Neurosci.

### 3.3. Comparison of Immune Function Indexes

Thirdly, we compared the immune function indexes of the two groups. The IL-6, IL-8, and IgE of the research group were lower compared to the control group, while the Th1/Th2 of the research group was higher compared to the control group, and the difference was statistically significant (*P* < 0.05). All the data results are indicated in Table 2.

### 3.4. Comparison of T Lymphocyte Subsets

Then, we compared the T lymphocyte subsets of the two groups, there exhibited no significant difference before nursing, but after treatment, the T lymphocyte subsets of the two groups decreased, and the levels of CD3+, CD4+, CD8+ and CD4+/CD8+ lymphocytes in the research group were lower compared to the control group, and the difference was statistically significant(*P* < 0.05). All the data results are indicated in Table 3.

### 3.5. Comparison of Physiological Function of Nasal Cavity

Next, we compared the nasal physiological function of the two groups, there exhibited no significant difference before treatment, but after treatment, the nasal physiological function of the two groups was enhanced, and the MTT, NR, and MCR of the research group were lower compared to the control group, and the difference was statistically significant (*P* < 0.05). The results of all the data are indicated in Table 4.

### 3.6. Comparison of the Incidence of Adverse Reactions

Finally, we compared the incidence of adverse reactions, the incidence of adverse reactions in the research group was lower compared to the control group, the difference was statistically significant, and the difference was statistically significant (*P* < 0.05). All the data results are indicated in Figure 2.

## 4. Discussion

AR is an inflammatory disease of the upper respiratory tract mediated by a variety of immune cells and IgE [14]. AR has become a global medical and health problem; studies indicate that the global incidence of AR patients is 10%–40%. AR seriously affects the work and life of patients and brings heavy economic pressure to individuals and society [14]. AR is difficult to cure and has a wide range of diseases. Its prevalence rate is as high as 10% to 20% in the world, which has had a great impact on the daily life of patients [15]. The prevalence rate of AR in mainland China has reached 4% and 38%, and has indicated an upward trend in recent years. The pathogenesis of AR is complex, and is caused by two main factors: heredity and environment, which leads to nasal mucosal inflammation. Allergen is the initiating factor of an allergic reaction, and lymphocytes, immune factors, and inflammatory reactions are important reasons for the progression of AR [16]. Under normal circumstances, the cellular physiology of the body dynamically maintains a state of balance, but when the balance is destroyed by the intervention of various inflammatory mediators and cytokines, the immune system is rapidly activated, which can lead to mucosal vasodilation and plasma exudation, resulting in a prolonged course of the disease and nasal mucosal tissue remodeling [17]. Therefore, it is generally believed that overactivation of the immune system and to allergy induced by IgE are the main reasons for the progress of AR [17]. This study explored the efficacy of different drugs combined with loratadine tablets in the treatment of AR and the effects of T lymphocyte subsets and nasal physiological function.

The article "Effect of Loratadine Tablets in Combination with Other Drugs on Nasal Physiological Function and T Lymphocyte Subsets in Patients with Allergic Rhinitis" was published in 2022. Journal: Comput Intell Neurosci.

In recent years, with the progress of society, especially in developed countries, air pollution is particularly serious. In the meantime, it has also become an important factor affecting AR. Qiong et al. pointed out that oak pollen exposure to SO2 and NO2 will lead to the destruction of its own structure and a significant increase in the number of pollen grains, thus increasing the prevalence of allergic airway diseases in sensitized individuals [18]. Some scholars have pointed out that there is a significant correlation between PM2.5 and PM10 and the prevalence of AR in adults. Total suspended particles, SO2, and NO2 in air pollutants are related to the increase in the prevalence of AR in children. Appropriate protective measures to the airway, such as wearing masks and reducing travel during pollen season, to reduce their exposure to air pollutants is an effective way to reduce the prevalence of AR. According to the severity of the patients, the corresponding standard drugs firstly should be taken, and the poor effect can be treated by further operation. Secondly, selective neurotomy, plasma ablation of the turbinate, and so on can be considered. Pterygoid canal neurotomy is a common surgical method. At present, Western medicine often employs AH, GC and other drugs or adjuvant immunity, desensitization, and other treatments, but its safety and side effects are still open to question, and it has the characteristics of a long course of treatment and high price [19].

At present, it is recognized that the pathogenesis of AR is closely related to the immune inflammatory response mediated by IgE. Studies have indicated that the disorder of immune response caused by the imbalance of Th1/Th2 in the body can induce the synthesis of IgE, which is the main cause of the disease. Meanwhile, the transformation of IL-4 secreted by Th2 can accelerate the absorption and infiltration of EOS, and the increase of sensitivity to allergic factors aggravates the clinical symptoms. The IgE antibody on the surface of MC on the nasal mucosa can also bind to IgE during the occurrence of AR, promote the release of LTs and a large number of inflammatory factors, and then accelerate the occurrence and development of AR [20]. Recent studies have also found that the pathogenic factors of AR are also related to the release of SP, VIP, and NPY neuropeptides released by inflammatory cells in vivo, which accelerate the release of EOS and aggravate the symptoms [20]. Western medicine mainly treats AR by GC, LTs (leukotriene), AH (antihistamine), and other drugs. In recent years, through the practice and research of clinical workers, the efficacy of these conventional medicine has been widely demonstrated [21]. However, it also has many defects, such as AH generally has a central inhibitory effect, external nasal use of GC is easy to cause drug-induced rhinitis, nasal decongestant use for a long time will make turbinate atrophy, drug response will increase, anticholinergic drugs will decrease with the aggravation of symptoms, and so on [21].

The article "Effect of Loratadine Tablets in Combination with Other Drugs on Nasal Physiological Function and T Lymphocyte Subsets in Patients with Allergic Rhinitis" was published in 2022. Journal: Comput Intell Neurosci.

The specific treatment of medicine can also be called desensitization therapy, mainly by improving the function of the body's immune system and weakening the overstimulation of external allergen reactions. it is an effective treatment for AR, which is divided into SLIT and SCIT [22]. The former is more easily accepted by patients, has more advantages in efficacy and safety, and is also suitable for children, while the latter can be used in combination with other drugs to achieve a better long-term effect. However, specific therapy also has some defects, such as too long treatment time, unstable curative effect, and long-term effective cooperation of patients.Chu et al. treated AR by blocking the nasal pterygoid canal, pharyngeal branch, and local ethmoid nerve [23]. However, most patients do not have a high degree of acceptance of surgical treatment, so they choose drug treatment.

Loratadine tablet is a tricyclic antihistamine with high efficiency and long-lasting effect, and it is a selective peripheral H1 receptor antagonist, which can relieve all kinds of symptoms caused by allergic reactions [24]. Antihistamines are available orally and intranasally. The first generation of antihistamine drugs such as chlorpheniramine and diphenhydramine is easy to cross the blood-brain barrier and bind to a large number of central H1 receptors, resulting in sedation, which is not recommended for clinical use [25]. In contrast, the second generation of antihistamines (cetirizine, levocetirizine, loratadine, desloratadine, and ebastine) can specifically bind to the peripheral H1 receptor and have a limited effect on permeating the blood-brain barrier, so it is safer. Glucocorticoid has a nonspecific anti-inflammatory effect. As a first-line drug in the clinical treatment of AR, glucocorticoid is mainly used in moderate and severe AR. It can effectively facilitate the nasal symptoms of children, but in the clinic, it is not easy for patients to master the correct spraying method and the use of antihormone drugs, and compliance is poor, which can easily lead to adverse reactions [26].

The article "Effect of Loratadine Tablets in Combination with Other Drugs on Nasal Physiological Function and T Lymphocyte Subsets in Patients with Allergic Rhinitis" was published in 2022. Journal: Comput Intell Neurosci.

Mometasone furoate nasal spray is one of the most commonly employed topical corticosteroids in the clinic [27]. It belongs to the third generation of nasal corticosteroids, which can not only play a good local anti-inflammatory effect but also be administered by nasal spray. can promote the drug to act directly on the nasal mucosa, thus can quickly and effectively alleviate the condition of children. In addition, studies have demonstrated that the combination of loratadine and loratadine is well tolerated, and mometasone furoate nasal spray has no significant effect on the plasma concentration of loratadine and its main metabolites [28]. Therefore, the use of mometasone furoate nasal spray combined with loratadine tablets in the treatment of children with AR can not only play a synergistic anti-inflammatory and antiallergic effect, so as to significantly facilitate the patient's condition and the level of inflammatory factors in the body. It can also facilitate the tolerance of patients to treatment. As a kind of glucocorticoid, budesonide is a locally effective anti-inflammatory drug. By inhibiting the release of inflammatory mediators, participate in the immune response of cytokines to achieve the purpose of treatment. Meanwhile, budesonide can protect against allergic reactions and prevent AR. The combination of the above two drugs can significantly facilitate the condition of patients with AR, enhance the effective rate of treatment, and promote the relief of clinical symptoms [29].

The changes in T lymphocytes play an important role in the occurrence and development of AR [30]. According to the cell surface differentiation antigen (CD), T lymphocytes are assigned into CD4+ and CD8+ subgroups and can be assigned into helper T cells (Th cells), and suppressor T cells (Ts cells) according to their functions. Therefore, the levels of T lymphocyte subsets and Th cell-related factors can reflect cellular immune status. In this study, budesonide and loratadine can significantly facilitate the changes of CD4+ and CD4+/CD8+ levels, and the levels of CD4+ and CD4+/CD8+ in the research group are significantly lower compared to the control group, indicating that budesonide and loratadine treatment can significantly facilitate the level of T lymphocyte subsets and avoid AR caused by overactivation of the immune system, which is consistent with the results reported by Germain et al. [30]. This is because budesonide and loratadine can reduce the excitability and sensitivity of parasympathetic nerves in sensitive areas of the nasal cavity, destroy nasal mucosa and weaken allergic reactions, so as to inhibit immune response and facilitate the level of T lymphocyte subsets [30]. Th cells can differentiate into Th1 and Th2, and the imbalance between these two cells will lead to the activation of immune-inflammatory factors and aggravate the local reaction in the nasal cavity, and lead to rhinitis. The production of IgE induced by the allergen is the main process leading to an allergic reaction, and IL-6 and IL-8 can stimulate the secretion of IgE by promoting the differentiation of acidic granulocytes. IL-6 and IL-8 can regulate the differentiation of Th cells and induce Th1/Th2 imbalance. Therefore, comparing the levels of IL-6 and IL-8 between the two groups can reflect the degree of immune response and inflammatory reaction. In this study, the two treatments could significantly affect the changes in IL-6 and IL-8 levels, and the levels of IL-6 and IL-8 in the research group were significantly lower compared to the control group, indicating that budesonide and loratadine could significantly reduce the levels of serum IL-6 and IL-8 in patients with AR, which was consistent with the results reported by Philipp et al. [31]. This is because budesonide and loratadine treatment can promote hyperemia to dilate vasoconstriction, contribute to tissue edema absorption, alleviate inflammatory response, and facilitate local immune status. Our study still has some shortcomings. Firstly, the quality of this study is limited due to the small sample size we included in the study. Secondly, this research is a single-center study and our findings are subject to some degree of bias. Therefore, our results may differ from those of large-scale multicenter studies from other academic institutes. Our research is still clinically significant and further in-depth investigations will be carried out in the future.

The article "Effect of Loratadine Tablets in Combination with Other Drugs on Nasal Physiological Function and T Lymphocyte Subsets in Patients with Allergic Rhinitis" was published in 2022. Journal: Comput Intell Neurosci.

In summary, compared with mometasone furoate nasal spray combined with loratadine tablets, budesonide and loratadine are more effective in the treatment of AR and can effectively improve the efficacy, T lymphocyte subsets and nasal physiological function of patients as well as with higher safety.

## Figures and Tables

**Figure 1:** Comparison of curative effect between two groups of patients.

**Figure 2:** Comparison of the incidence of adverse reactions between two groups of patients.

**Table 1:** Comparison of clinical symptom relief time between the two groups [$\bar{x}\pm s$, *d*].

Grouping	*N*	Nasal congestion	Nasal itching	Runny nose	Sneeze
Control group	60	5.94 ± 0.41	5.89 ± 0.67	6.98 ± 0.67	6.45 ± 0.41
Research group	60	4.19 ± 1.22	4.16 ± 0.34	4.33 ± 0.31	4.10 ± 0.35
*t* value		10.532	17.835	27.805	33.767
*P* value		<0.01	<0.01	<0.01	<0.01

**Table 2:** Comparison of immune function indexes between the two groups [$\bar{x}\pm s$].

Grouping	*N*	IL-6 (pg/ml)	IL-8 (ng/l)	IgE (IU/ml)	Th1/Th2
Control group	60	56.34 ± 3.21	90.94 ± 1.42	67.94 ± 1.24	1.01 ± 0.44
Research group	60	50.94 ± 3.11	83.43 ± 1.22	54.91 ± 1.22	1.15 ± 0.23
*t* value		9.358	31.073	58.021	2.184
*P* value		<0.01	<0.01	<0.01	<0.01

**Table 3:** Comparison of T lymphocyte subsets between the two groups [$\bar{x}\pm s$].

Grouping	*N*	CD3＋(%)	CD4＋(%)	CD8＋(%)	CD4＋/CD8＋
Control group	60	68.94 ± 1.22	38.95 ± 3.11	24.34 ± 0.66	1.78 ± 0.42
Research group	60	65.29 ± 1.35	33.65 ± 3.15	22.85 ± 1.21	1.42 ± 0.21
*t* value		15.538	15.538	8.373	5.938
*P* value		<0.01	<0.01	<0.01	<0.01

**Table 4:** Comparison of physiological function of nasal cavity between the two groups [$\bar{x}\pm s$].

Grouping	*N*	MTT (min)		NR (Pa/cm^3^·s)		MCR (mm/min)	
		Before treatment	After treatment	Before treatment	After treatment	Before treatment	After treatment
Control group	60	21.53 ± 3.31	17.39 ± 3.34	0.29 ± 0.06	0.19 ± 0.03	7.78 ± 1.23	5.39 ± 0.16
Research group	60	21.95 ± 3.34	13.81 ± 2.14	0.28 ± 0.01	0.14 ± 0.05	7.72 ± 1.26	4.12 ± 0.31
*t* value		0.691	6.990	1.273	6.642	0.263	28.199
*P* value		>0.05	<0.01	>0.05	<0.01	>0.05	<0.01

## Data Availability

The datasets used and analyzed during the current study are available from the corresponding author upon reasonable request.
